# Characterization of a Novel Chromatin Sorting Tool Reveals Importance of Histone Variant H3.3 in Contextual Fear Memory and Motor Learning

**DOI:** 10.3389/fnmol.2016.00011

**Published:** 2016-02-09

**Authors:** Anna G. McNally, Shane G. Poplawski, Brittany A. Mayweather, Kyle M. White, Ted Abel

**Affiliations:** ^1^Pharmacology Graduate Group, University of PennsylvaniaPhiladelphia, PA, USA; ^2^Department of Biology, University of PennsylvaniaPhiladelphia, PA, USA

**Keywords:** histone variant, epigenetics, excitatory neuron, hippocampus, memory consolidation

## Abstract

The consolidation of short-term labile memories for long-term storage requires transcription and there is growing interest in defining the epigenetic mechanisms regulating these transcriptional events. In particular, it has been hypothesized that combinations of histone post-translational modifications (PTMs) have the potential to store memory by dynamically defining the transcriptional status of any given gene loci. Studying epigenetic phenomena during long-term memory consolidation, however, is complicated by the complex cellular heterogeneity of the brain, in which epigenetic signal from memory-relevant cells can be obscured or diluted by the surrounding milieu. To address this issue, we have developed a transgenic mouse line expressing a tetO-regulated, hemagglutinin (HA)-tagged histone H3.3 exclusively in excitatory neurons of the forebrain. Unlike canonical histones, histone H3.3 is incorporated at promoter regions of transcriptionally active genes in a DNA replication-independent manner, stably “barcoding” active regions of the genome in post-mitotic cells. Immunoprecipitating H3.3-HA containing nucleosomes from the hippocampus will therefore enrich for memory-relevant chromatin by isolating actively transcribed regions of the excitatory neuron genome. To evaluate the validity of using H3.3 “barcoding” to sort chromatin, we performed a molecular and behavioral characterization of the H3.3-HA transgenic mouse line. Expectedly, we find that H3.3-HA is incorporated preferentially at promoter regions of actively-transcribed neuronal genes and that expression can be effectively regulated by doxycycline. Additionally, H3.3-HA overexpression does not adversely affect exploratory or anxiety-related behaviors, nor does it affect spatial memory. Transgenic animals do, however, exhibit deficits in contextual memory and motor learning, revealing the importance of this histone isoform in the brain. Future studies in the H3.3-HA transgenic mouse line will define the combinatorial histone PTM landscape during spatial memory consolidation and will investigate the important contributions of histone H3.3 to the normal functioning of the brain.

## Introduction

It is a fundamental goal in neuroscience to understand the mechanisms that regulate the formation of long-term memory. Short-term labile memories are consolidated for long-term storage through a transcription-dependent process known as memory consolidation (Agranoff et al., 1967; Nguyen et al., 1994). Although the requirement for transcription to stabilize short-term memories was demonstrated decades ago, the epigenetic processes regulating this transcription are only beginning to be uncovered. Histone post-translational modifications, or PTMs, are one such epigenetic phenomenon thought to be critical to the regulation of gene expression during long-term memory consolidation. Indeed, many modifications correlate with transcriptional level (Wang et al., 2008). Notably, histone acetylation contributes to an active transcriptional state and is critical for both long-term memory and pharmacological memory enhancement (Levenson et al., 2004; Vecsey et al., 2007; Bousiges et al., 2010; Peleg et al., 2010; Park et al., 2013; Dagnas et al., 2015).

While significant advances have been made in understanding the contributions of individual histone PTMs to long-term memory, current models postulate that histone acetylation and other PTMs function in a combinatorial fashion to dynamically regulate gene expression through alterations in chromatin accessibility and guiding the association of chromatin-binding proteins to specific genetic loci (Jenuwein and Allis, 2001; Berger, 2007). Identifying changes in the histone PTM landscape within the brain, however, is complicated by the presence of a complex cellular milieu. Long-term memory is thought to depend critically on transcriptional changes within excitatory neurons, yet epigenetic signal occurring within these cells will likely be obscured or diluted by surrounding cell types (Kauer et al., 1988; Tocco et al., 1991). Currently, few tools exist to study chromatin from within specific cellular populations. Fluorescence-activated cell sorting (FACS) is perhaps the most widely used sorting approach, but this technique is labor-intensive and has the potential to disrupt chromatin dynamics and gene expression (Jiang et al., 2008). There is therefore a substantial need for a simple approach which can be adapted to multiple cell types.

For these reasons, we have developed a transgenic mouse line expressing a tetO-regulated hemagglutinin (HA)-tagged histone variant, known as H3.3, specifically within excitatory neurons of the forebrain. Unlike canonical histones, histone H3.3 is incorporated at promoters of transcriptionally active genes in a DNA replication-independent manner, effectively “barcoding” active regions of the genome (Ahmad and Henikoff, 2002; Chow et al., 2005; Mito et al., 2005; Daury et al., 2006; Hake and Allis, 2006). By combining the tetO-regulated tagged histone with the tetracycline transactivator system, we can control both the temporal and spatial regulation of transgene expression. Here, we employ the CaMKIIα-tTA driver line to express the tagged histone H3.3 specifically in excitatory forebrain neurons, and limit its expression to adulthood by administering doxycycline in the diet (Mayford et al., 1996). Chromatin immunoprecipitation (ChIP) for the HA tag can then isolate nucleosomes bound to active regions of the excitatory neuron genome, greatly enriching for those regions most likely to be altered during long-term memory consolidation. Mass spectrometry could then be employed to define the histone PTM landscape occurring in response to learning (Young et al., 2009; Britton et al., 2011). In the current study, we perform a molecular and behavioral characterization of the H3.3-HA transgenic mouse line to evaluate the validity of this chromatin sorting approach.

## Materials and Methods

### Subjects

To create tetO-H3.3-HA mice, a mouse-codon optimized N-terminal tagged H3.3-HA sequence from GeneArt (Thermo Fisher Scientific) was cloned into the MM400 plasmid containing the tetO tetracycline-regulatable enhancer element, as previously described (Hawk et al., 2012). The plasmid was digested using Not1 (New England Biolabs #R0189S) and the 2.5-kb tetO-H3.3-HA transgene fragment was sequenced to ensure complete sequence accuracy. The gel-purified transgene was submitted to the Transgenic and Chimeric Mouse Facility at the University of Pennsylvania, where it was injected into C57BL/6J pronuclei. Mice were genotyped by Southern Blotting using transgene-specific primers (F: GCGTCCATCTGGTCAGAAA, R: TGGAATCTCAGGTCGGTCTT). Four founder lines were generated and crossed with C57BL/6J mice expressing the CaMKIIα-tTA transgene (Mayford et al., 1996). Double-transgenic males (CaMKIIα-tTA+; tetO-H3.3-HA+) from the highest expressing line were chosen for active breeding to C57BL/6J females (The Jackson Laboratory). Non-transgenic and single-transgenic littermates served as wildtype controls. Mice were bred and raised on doxycycline chow until weaning (unless otherwise noted) to restrict transgene expression to adulthood.

Adult transgenic and control mice were group housed on a 12:12 light:dark cycle, with food and water access *ad libitum*. Behavioral experiments were conducted during the light cycle between 7 and 10 am. All experiments were approved by the Institution of Animal Care and Use Committee of the University of Pennsylvania and conducted in accordance with the National Institutes of Health guidelines.

### Immunostaining

Anesthetized double-transgenic and wildtype littermates were transcardially perfused with 4% PFA using a peristaltic perfusion pump (Rainin Instruments). Thirty micrometer (30 μM) coronal sections were then collected in PBS, permeabilized in 0.1% Triton X-100 for 5 min, quenched in 1% H_2_O_2_ for 15 min, and blocked in 8% normal goat serum (NGS) containing 0.3% Triton X-100 for 50 min at RT. The following incubation steps were then performed with intervening PBS washes (3 × 5 min each): HA antibody (1:500, Roche Clone 3F10) in 2% NGS and 0.3% Triton X-100 overnight at 4°C, biotinylated goat anti-rat antibody (1:1000, Jackson ImmunoResearch #112-065-003) in PBST for 2 h at RT, Vectastain ABC solution (Vector Laboratories #PK-4000) for 1.5 h at RT, DAB solution (0.2 mg/ml) containing 0.005% H_2_O_2_ for 20 min at RT. Sections were then washed in PBS containing 0.01% sodium azide and mounted in 0.7% gelatin. Mounted sections were counterstained with 0.1% cresyl violet acetate (where indicated), coverslipped, and visualized through a light microscope.

For immunofluorescence staining, 30 μM sections were permeabilized and blocked as before and then incubated at 4°C overnight using the following primary antibodies: HA (1:500, Roche Clone 3F10), CaMKIIα (1:1000, Santa Cruz #sc-32288), Gfap alexafluor 488-conjugated (1:1000, Millipore #MAB3402X), and Pvalb (1:1000, Abcam #ab11427). Sections were then washed in PBS followed by the addition of DAPI (Thermo Fisher Scientific #R37605) and the respective secondary antibody: goat anti-rat Alexa Fluor 555 for HA (1:1000, Invitrogen #A-21434), goat anti-mouse Alexa Fluor 488 for CaMKIIα (1:000, Invitrogen #A-11001), and goat anti-rabbit Alexa Fluor 488 for Pvalb (1:1000, Invitrogen #A-11034). Sections were incubated in the dark for 2 h at RT, washed in PBS, mounted, dried overnight at 4°C, and coverslipped using PermaFluor Mounting Medium (Thermo Fisher Scientific #TA-030-FM). Images were collected using a Leica Widefield Microscope.

### Chromatin Immunoprecipitation (ChIP)

Hippocampi were dissected from double- and single- transgenic mice and finely cut using a razor blade. Fragments were incubated in 2% PFA for 10 min at RT, followed by the addition of 100 μl 1M glycine to quench the reaction. ChIP was performed as previously described (Vecsey et al., 2007). Briefly, tissue was dounce homogenized and the nuclei lysed. Chromatin was then sheared using a Bioruptor (Diagenode) with two 15-min cycles of 1 min on and 1.5 min off. IP samples were incubated with 2 μg HA antibody (Roche Clone 3F10) at 4°C overnight. The following day, samples were incubated in a 50% slurry of Protein G Agarose beads (Pierce #20398) for 2 h at 4°C. Beads were washed in low salt buffer, high salt buffer, LiCl buffer, and twice in 1X TE buffer. DNA was then eluted at RT in 200 μl ChIP elution buffer (1% SDS/0.1M NaHCO_3_). IP and input control samples were reverse-crosslinked at 65°C overnight in 200 mM NaCl, followed by treatment with proteinase K for 1 h at 55°C. DNA was purified using the Qiagen Qiaquick PCR Purification Kit and eluted in 200 μl water.

### Quantitative RT-PCR (qPCR)

Reactions were performed in 384 well plates using the Viia7 Real Time PCR System (Applied Biosystems). Reactions consisted of 2.5 μl Fast SYBR Green Master Mix (Thermo Fisher Scientific #4385614), 0.25 μl 5 μM primer mix, and 2.25 μl ChIP or input DNA, performed in quadruplicate. The following primers were used (5′ to 3′): *Nr4a1* (F: GGAGCCTAGTGGGTCTGGAAGC, R: GGAGCGCGGATTGTTTGATCT), *Nr4a2* (F: GGGCTTGGGGGCGATGGTTC, R: AGGATCCGGCAACAGGTGCG), *Nr4a3* (F: GAGGGAGGAGGAGGGTGACGTA, R: CATAGAGTGCCTGGAATGCGAGA), *Snap25* (F: AGCCCCGGGCAAACAACTCG, R: TTGGGTTTGCAGGGCTAGGGC), *Gfap* (F: GCTGTTCCCTCGGCCCTCTCT, R: CACCAGCCTGGCTTCGCCAT), *Olig2* (F: AGGGAGTGGGGGCCTTCTGC, R: CCTCCTGTTTCCCGCTGCCG), *Apcs* (F: AGACCCAGCTGCAGAATGGAGA, R: TGCTGGGAAGGGAAGAGCTGC), *Fgb* (F: ACGAGACCTCCGAGACAGGGC, R: TGTGGACACAGGGGGTTCCTCG), *Line1* (F: AACGAGGAGTTGGTTCTTTGAG, R: TTTGTCCCTGTGCCCTTTAGTGA), *Snap25 5′ UTR* (F: CAGCAGCCTCCATGCCCCAC, R: CTGAGCTCCCGCCATCGCAC), *Snap25 3′ UTR* (F: ACGCATGCTCAGTATTGGGACACT, R: ACACAGCTGCAGGTTTTGCTGGT), *Snap2*5 T*ES* (F: TCACACCAGAAAACACAGTCTGCAT, R: ACCAAGCCAAAGTGTCCATTGTCAT), *Nr4a*1 E*xon1* (F: TCTGGACGCACCCGTGACCT, R: CCCTCGCTGCCACCTGAAGC), *Nr4a*1 T*ES* (F: GGACAGCGGCTAACCCAGGGA. R: ACCTGAGACCCAAGGCCAGGTC). Data were normalized as percent input and to repeat element *Line1*. Fold change of double- to single-transgenic mice was determined and fold changes were compared using unpaired *t*-tests, with two-tailed *p* values reported.

### Behavioral Procedures

Two cohorts of double-transgenic and wildtype male mice (aged 3–4 months) were used for behavioral testing, with two additional cohorts kept continuously on doxycycline (Bio-Serv, 40 mg/kg) for behavioral rescue experiments. Wildtype mice included both single-transgenic and non-transgenic littermates. The behavioral tasks were performed in the following order with at least 1 week recovery between tasks: Rotarod, open field, object location memory (OLM), and contextual fear conditioning. Weights were recorded in male mice prior to the rotarod task. Mice were group housed until 1 week prior to contextual fear training, at which point animals were housed individually. Female mice (aged 3–4 months) were evaluated in rotarod, open field, and contextual fear conditioning.

#### Rotarod

The rotarod apparatus contains a rotating rod (3 cm diameter) raised 16 cm above a platform, divided into five sections. The rotarod task was performed as previously described (Oliveira et al., 2006). Briefly, on habituation day, mice were placed on the rod rotating at 4 RPM for 30 s. The following three consecutive days consisted of testing trials, where mice underwent three 5 min trials per day, with an inter-trial interval of 1 h. During testing trials, the rotarod gradually accelerated from 4 to 40 RPM over the course of 5 min. Latency to fail was recorded, with failure defined as falling off or passively gripping onto the rod. A repeated measures ANOVA was used to compare latencies to fail across testing sessions. Bonferroni correction was used to adjust for multiple comparisons.

#### Open Field

Locomotor activity was measured for 30 min in a 41 × 41 cm Open Field (San Diego Instruments). The box was equipped with a 16 × 16 photobeam configuration, spaced every 2.54 cm. Total ambulation and preference for the periphery vs. the center of the open field were measured by number of beam breaks (Stein et al., 2006) and group means were compared across genotypes using unpaired *t*-tests, with two-tailed *p* values reported.

#### Object Location Memory (OLM)

Mice were handled in the experimental setting for five consecutive days (5 min/mouse) prior to OLM training. Training and testing were performed as previously described (Havekes et al., 2014) and both began at lights on (7 am). On training day, mice were placed individually into the training arena which contained an internal visual cue on one of the four walls. Mice underwent a total of four 6 min sessions, with an intersession interval of 3 min in the home cage. The first session consisted of habituation to the empty arena, while the following three sessions contained three distinct objects (a glass bottle, metal tower, and plastic cylinder). Arenas and objects were wiped down between all sessions with 70% ethanol. Twenty-four hours following training, mice were re-exposed to the arena for 6 min, with one object displaced to a novel spatial location. Training and testing sessions were video monitored and object exploration times were scored off-line by an experimenter blind to genotype. OLM was assessed by calculating the percent preference for the displaced object relative to all objects (DO/(DO + NDO) during testing. A two-way ANOVA was used to compare training and testing means, with Tukey’s *post hoc* analysis performed where indicated. A repeated measures ANOVA was used to compare exploration time across the three training sessions. Bonferroni correction was used to adjust for multiple comparisons.

#### Contextual Fear Conditioning

Individually housed double-transgenic and wildtype mice were handled for three consecutive days (1 min/mouse) prior to contextual fear training. Handling occurred in the same experimental setting without context exposure. Training and testing were performed as previously described (Wood et al., 2006; Vecsey et al., 2007; Hawk et al., 2012). The training session entailed a single 2 s, 1.5 mA foot shock, terminating 2.5 min after placement of the mouse in the chamber (Med-Associates, 31.8 × 25.4 × 26.7 cm). The mouse remained in the chamber for an additional 30 s and was then returned to the homecage. A 5 min test session was conducted 24 h following training where the mouse was re-exposed to the context in the absence of a footshock. Freezing behavior was measured during all sessions using automated scoring software (Clever Systems). Multiple unpaired *t*-tests were used to compare pre-shock and 24 h test freezing levels between genotypes, with multiple comparison adjustments made using the Holm-Sidak method.

### Statistical Analyses

All data are presented as mean ± SEM and analyzed using GraphPad Prism 6 software. Comparisons were made using unpaired *t*-tests, two-way ANOVA, or two-way repeated measures ANOVA, as indicated. *Post hoc* tests were used where appropriate. For all statistical tests, *p* < 0.05 was considered significant.

## Results

### Novel Sorting Strategy for the Isolation of Active Chromatin from Excitatory Neurons

In this study, founder lines expressing a tetO-regulated HA-tagged histone H3.3 in C57BL/6J mice were generated and crossed with an excitatory neuron-specific tetracycline transactivator (tTA) line, CaMKIIα-tTA (Mayford et al., 1996) to produce double-transgenic mice (Figure 1A). Histone variant H3.3 was selected because it is known to incorporate at promoters of transcriptionally active genes in a DNA replication-independent manner, effectively “barcoding” active regions of the genome (Hake and Allis, 2006). By combining tagged H3.3 with the tetracycline-transactivator system, standard chromatin immunoprecipitation methodologies can be employed to enrich for active regions of the excitatory neuron genome in the mouse hippocampus during behavioral tasks.

**Figure 1:** **Tagging histone H3.3 in excitatory neurons of the forebrain as a novel epigenetic tool to sort chromatin. (A)** CaMKIIα-tTA transgene was used to drive expression of the tetO-regulated HA-tagged histone H3.3 exclusively in excitatory neurons of the forebrain. **(B)** In double-transgenic mice, DAB staining for the HA tag revealed robust expression of H3.3-HA in the hippocampus, striatum, and cortex, but not in the cerebellum. **(C)** Double-transgenic mice removed from a doxycycline diet at weaning displayed high expression of H3.3-HA (brown), while mice receiving continuous doxycycline showed no expression. Cresyl violet was used as a counterstain. **(D)** Hippocampal immunofluorescent staining divided into green channel (1st panel), red channel (2nd panel), blue channel (3rd panel) and overlay (4th panel). H3.3-HA colocalizes exclusively with excitatory neuron marker CaMKIIα, and not astrocyte marker Gfap, or inhibitory neuron marker Pvalb. (CaMKIIα = Ca^2+^/calmodulin-dependent protein kinase II; Gfap = glial fibrillary acidic protein; Pvalb = parvalbumin).

### H3.3-HA Expression is Restricted to Excitatory Neurons of the Forebrain

The first step in validating the feasibility of this approach was to demonstrate the expected expression patterns of H3.3-HA. As anticipated, immunostaining for the HA tag in double-transgenic and wildtype littermates revealed pronounced expression of H3.3-HA in areas of the forebrain, including the hippocampus, striatum, and cortex, with no expression observed in the cerebellum (Figure 1B). Exploiting one of the key advantages of the tetracycline transactivator system, we next wanted to determine if transgene expression could be controlled through the administration of doxycycline in the diet (Bio-Serv, 40 mg/kg). Indeed, mice removed from doxycycline at weaning (postnatal day 28) showed marked H3.3-HA expression at postnatal day 60, particularly in the dentate gyrus (Figure 1C). In contrast, mice that remained on a doxycycline diet showed no transgene expression. Restricting transgene expression to adulthood in this way avoided potentially confounding effects of H3.3-HA overexpression on development.

Finally, we wanted to demonstrate that H3.3-HA expression was specific to excitatory neurons expressing CaMKIIα in the hippocampus. Using immunofluorescent staining to compare the overlay of the HA tag and DAPI counterstain with CaMKIIα, Gfap (astrocyte marker), and Pvalb (inhibitory neuron marker), we found that H3.3-HA colocalized exclusively with excitatory neurons, and was not expressed in glia or inhibitory neurons (Figure 1D). Colocalization was nearly complete in the dentate gyrus, particularly within the subgranular zone (Figure 1D). Together, these findings suggest that ChIP of the HA tag from hippocampal tissue should selectively isolate only chromatin from excitatory neurons.

### Chromatin Immunoprecipitation of H3.3-HA Isolates Active Regions of the Excitatory Neuron Genome

Based on the known incorporation of histone variant H3.3 into regions of active transcription, we expected that ChIP of the HA tag would enrich for genomic regions that are actively transcribed in excitatory neurons. Indeed, immunoprecipitating chromatin containing H3.3-HA from whole hippocampi showed enrichment for promoters of genes expressed in excitatory neurons (*Nr4a1, Nr4a2, Nr4a3, Snap25*), over genes expressed specifically in glial (*Gfap, Olig2*) or liver cells (*Apcs, Fgb*; Figure 2A). The nuclear receptor 4a (*nr4a*) family of transcription factors are activity-dependent CREB target genes that are critical effectors of long-term memory (Bridi and Abel, 2013). Synaptosomal-associated protein 25 (*snap25*) is a neuron-specific SNARE protein that mediates synaptic vesicle membrane docking and fusion (Oyler et al., 1989). Enrichment at non-neuronal genes was evaluated using astrocyte-specific gene, glial fribrillary acidic protein (*gfap*), a key mediator of astrocyte-neuron interactions, and oligodendrocyte-specific gene, oligodendrocyte lineage transcription factor 2 (*olig2*), a transcription factor required for oligodendrocyte determination (Weinstein et al., 1991; Brenner et al., 1994; Takebayashi et al., 2002). Two liver-specific genes were used as controls, serum amyloid P component (*apcs*) and fibrinogen beta chain (*fgb*), as these genes are not expressed in the brain (Peixoto et al., 2015).

**Figure 2:** **ChIP for H3.3-HA enriches for promoters of genes active in excitatory neurons. (A)** ChIP was performed for the HA tag of H3.3-HA from whole hippocampi and primers against promoters of neuron-, astrocyte-, oligodendrocyte-, and liver- specific genes were evaluated. Neuronally-expressed genes were significantly more enriched over genes expressed in other cell types. **(B)** Primers were selected throughout two neuronally expressed genes. Enrichment was biased toward the promoter of both genes tested as compared to transcription end sites (TES) and untranslated regions (UTR). Data are presented as mean fold enrichment over single-transgenic controls ± SEM (*n* = 3 per group). *p < 0.05. (*nr4a* = nuclear receptor 4a; *snap25* = synaptosomal-associated protein 25 kda; *olig2* = oligodendrocyte transcription factor 2; *apcs* = amyloid P component, serum; *fgb* = fibrinogen beta chain).

Additionally, because H3.3 has exhibited promoter bias in other systems (Chow et al., 2005), we next wanted to test if H3.3-HA was preferentially incorporated at promoters of neuronally-expressed genes as compared to gene bodies. Using primers specific to these regions in two neuronally expressed genes, we found that gene promoters had the highest proportion of H3.3-HA incorporation (Figure 2B). These data suggest that this sorting strategy will enrich for promoters of genes specifically expressed in excitatory neurons. This tool could therefore be useful not only for isolating active regions of the excitatory neuron genome, but also for studying the incorporation of H3.3 throughout the genome during learning; a currently nascent area of research (Maze et al., 2015).

### Overexpression of H3.3-HA in Excitatory Neurons of the Forebrain does not Affect Exploration, Anxiety-Related Behavior, or Spatial Memory

An important next step in the characterization of this novel tool was to test the performance of these animals in a battery of behavioral tasks, as abnormalities in specific behaviors have been observed in other overexpressing tagged histones (Ito et al., 2014). In the open field paradigm, mice are allowed to explore a novel, enclosed open field for 30 min, with locomotor activity assessed through the automatic scoring of beam breaks (Stein et al., 2006). No difference in total ambulation was detected between transgenic mice and their wildtype littermates (*p* = 0.195), indicating that exploratory behavior is unaffected by H3.3-HA overexpression (Figure 3A). This result was corroborated in female mice (*p* = 0.667). In comparing preference for the periphery of the open field vs. the center, both genotypes displayed a marked preference for the periphery of the open field, as expected, with no difference in percent center activity between genotypes (*p* = 0.494; Figure 3B). Percent center activity was similarly comparable between genotypes in female mice (*p* = 0.924). This indicates an absence of gross anxiety-related deficits in the double-transgenic animals.

**Figure 3:** **Overexpression of H3.3-HA in excitatory neurons of the forebrain does not affect exploration, anxiety-related behavior, or spatial memory. (A)** There was no difference in total ambulation (as measured by beam breaks) between genotypes across 30 min of exploration in an open field. **(B)** Double-transgenic and wildtype mice exhibited a comparable preference for the periphery of an open field vs. the center (*n* = 9–11 per group). **(C)** Schematic diagram illustrating the object-location memory (OLM) task during habituation (left), training (middle) and testing (right). Testing was performed 24 h after training. Both genotypes showed a decrease in total object exploration time during the three consecutive training sessions, as expected. **(D)** Double-transgenic and wildtype mice exhibited a comparable and significant preference for the displaced object during testing as compared to training, signifying long-term object-location memory. Preference for the displaced object was calculated as the percentage of object exploration time dedicated to this object as compared to all objects (DO/(DO + NDO). Dotted line indicates chance performance. Data are presented as group means ± SEM (*n* = 18 per group). *p < 0.05.

This sorting tool was developed to study the epigenetic changes occurring in active regions of the excitatory neuron genome during long-term memory consolidation. Accordingly, we wanted to evaluate the performance of these animals in memory tasks. In the OLM task (OLM), mice explore an arena containing three distinct objects arranged in a specific spatial orientation. The following day, mice are re-exposed to the same arena, but with one object displaced to a novel spatial location. Long-term spatial memory is then assessed by measuring the preference for the displaced object as compared to all objects at testing (Havekes et al., 2014). Across all three training sessions, both double-transgenic mice and their wildtype littermates showed a comparable decrease in total object exploration time (*F*_(2,68)_ = 22.13, *p* < 0.0001), with no effect of genotype (*F*_(1,34)_ = 1.36, *p* = 0.25) or a training session × genotype interaction observed (*F*_(2,68)_ = 0.84, *p* = 0.44; Figure 3C). Both genotypes also displayed a significant preference for the displaced object during testing (*F*_(1,68)_ = 29.64, *p* < 0.0001) as compared to training, indicating intact long-term spatial memory (Figure 3D). No effect of genotype (*F*_(1,68)_ = 0.988, *p* = 0.32) or a session × genotype interaction was observed (*F*_(1,68)_ = 0.031, *p* = 0.86).

### Double-Transgenic Mice have Deficits in Contextual Fear Memory and Motor Learning

In contrast to OLM, the contextual fear conditioning task has the advantage of allowing for the precise temporal resolution of the molecular events occurring in the hippocampus during a learning event, as only a single training session is required to develop a robust contextual memory (Bourtchouladze et al., 1998). For this reason, contextual fear conditioning would be the preferred paradigm to use in conjunction with this novel chromatin sorting tool. In this task, long-term retention of a context-shock association is evaluated by measuring freezing behavior (Wood et al., 2006; Vecsey et al., 2007; Hawk et al., 2012). Interestingly, while both double-transgenic and wildtype mice displayed a significant increase in freezing behavior at the 24 h test as compared to pre-shock freezing levels (*t* = 3.51, *p* = 0.001; *t* = 8.67, *p* < 0.0001, respectively), demonstrating the capacity for contextual learning, double-transgenic mice froze at significantly lower levels than their wildtype littermates at the 24 h test (*t* = 2.86, *p* = 0.007; Figure 4A). Similarly in females, both genotypes showed increased freezing behavior at the 24 h test as compared to pre-shock levels (*t* = 2.99, *p* = 0.008; *t* = 4.48, *p* = 0.002), with double-transgenic mice freezing at significantly lower levels than their wildtype littermates at the 24 h test (*t* = 3.83, *p* = 0.002).

**Figure 4:** **Overexpression of H3.3-HA in excitatory neurons of the forebrain induces deficits in contextual fear memory and motor learning. (A)** While both genotypes displayed significant increases in percent freezing at the 24 h test as compared to pre-shock levels, double-transgenic mice froze at significantly lower levels than their wildtype littermates at the 24 h test (*n* = 17–18 per group). **(B)** Across testing days, there was a significant improvement in time spent on the rotating rod for both genotypes. Despite comparable latencies to fail on testing day 1, double-transgenic mice displayed significantly lower latencies to fail on testing days 2 and 3, indicating deficits in motor learning. Data are presented as group means ± SEM (*n* = 10–11 per group). *p < 0.05.

In addition to memory tasks, we also wanted to evaluate motor learning using the rotarod task. In this task, mice are placed on a slowly-accelerating rod and latencies to fail are measured across three testing session (Oliveira et al., 2006). Prior to rotarod testing, body weights were evaluated. No difference was observed between double-transgenic and wildtype mice (*p* = 0.12). Both double-transgenic and wildtype mice exhibited a significant improvement in time spent on the rotating rod across testing sessions (*F*_(2,38)_ = 28.34, *p* < 0.0001). Despite comparable latencies to fail on test day 1, double-transgenic mice had significantly lower latencies to fail on testing days 2 and 3 than their wildtype littermates (*F*_(1,19)_ = 12.66, *p* = 0.0021), indicating deficits in motor learning. No effect of genotype × trial day interaction was observed (*F*_(2,38)_ = 0.96, *p* = 0.39; Figure 4B). In female mice, both genotypes significantly improved in time spent on the rotating rod across trials (effect of trial *F*_(2,24)_ = 16.46, *p* < 0.0001). In contrast to male mice, female double-transgenic mice had significantly lower latencies to fail only on testing day 1 (effect of genotype *F*_(1,12)_ = 5.76, *p* = 0.0335. This may suggest deficits in motor coordination, as opposed to motor learning. No effect of genotype × trial interaction (*F*_(2,24)_ = 2.39, *p* = NS) was observed.

### Doxycycline Rescues Deficits in Contextual Fear Conditioning and Rotarod

To determine if the observed behavioral deficits were a direct result of H3.3-HA overexpression, or were simply an effect of transgene insertion, two cohorts of male double-transgenic and wildtype mice were kept continuously on doxycycline to suppress H3.3-HA expression. Despite the double-transgenic animals having significantly higher pre-shock freezing levels (*t* = 2.35, *p* = 0.027), both genotypes displayed significant increases in percent freezing at the 24 h test as compared to pre-shock levels (*t* = 6.35, *p* < 0.0001; *t* = 6.13, *p* < 0.0001, respectively), indicating a learned association between context and shock. Importantly, doxycycline fully rescued the deficits in freezing levels observed in the transgenic animals at the 24 h test (*t* = 1.31, *p* = 0.20), implicating H3.3-HA overexpression as driving impairments in contextual fear memory (Figure 5A).

**Figure 5:** **Doxycycline rescues deficits in contextual fear memory and motor learning. (A)** Both genotypes exhibited significant increases in percent freezing at the 24 h test as compared to pre-shock levels. There was no statistical difference in percent freezing at the 24 h test between genotypes (*n* = 13 per group). **(B)** Across testing days, both genotypes exhibited a significant improvement in time spent on the rotating rod, and performance was comparable on all days (*n* = 6–8 per group). Data are presented as group means ± SEM. *p < 0.05.

We next wanted to test whether this rescue effect could be extended to the rotarod task. Indeed, across testing days, both genotypes exhibited a significant improvement in time spent on the rotating rod (*F*_(2,24)_ = 10.28, *p* = 0.0006) with no effect of genotype (*F*_(1,12)_ = 0.48, *p* = 0.50) or a genotype × trial day interaction (*F*_(2,24)_ = 0.21, *p* = 0.81) observed (Figure 5B).

## Discussion

Despite significant advances in the field of neuroepigenetics, studying epigenetic phenomenon is complicated by the complex cellular heterogeneity of the brain. Currently, few tools exist to examine epigenetic regulation in specific cellular populations. Prior attempts to perform epigenetic analysis in a cell-type specific manner have used FACS, but this technique relies on harsh separating techniques that have the potential to alter the epigenome (Jiang et al., 2008). In the present study, we employ a novel tool based on histone H3.3 “barcoding” to isolate actively transcribed regions of the excitatory neuron genome using standard ChIP protocols (Hake and Allis, 2006). We create transgenic mice that express the tagged histone exclusively in excitatory neurons of the forebrain in a doxycycline-regulatable manner. Importantly, we find that ChIP for H3.3-HA isolates promoters of genes active in excitatory neurons over genes expressed in other cell types, demonstrating that H3.3-HA is effectively marking active regions of the genome. In addition to a molecular characterization, we also evaluated the performance of the transgenic animals in several behavioral tasks, as genetic alterations in the brain have the potential to alter behavior (Leach et al., 2012; Cao et al., 2014; Ito et al., 2014). We find that H3.3-HA overexpression does not alter exploratory or anxiety-related phenotypes and does not interfere with long-term spatial memory. Transgene expression does, however, cause deficits in contextual memory and motor learning; effects that can be rescued by the continuous administration of doxycycline in the diet. Collectively, these findings establish the validity of employing histone “barcoding” to sort active regions of the excitatory neuron genome. We anticipate that this technique will be useful in studying the epigenome during spatial memory consolidation.

One often overlooked aspect in the characterization of new transgenic mouse lines is the effect of transgene expression on behavior. Indeed, there are many examples of unexpected consequences of transgene overexpression in the brain (Gong et al., 2011; Ito et al., 2014). By using behavioral tasks with known neural correlates, we can start to delineate which brain regions are most sensitive to H3.3-HA overexpression. Contextual fear conditioning is known to require both the amygdala and the hippocampus, while OLM is dependent on the hippocampus (Phillips and LeDoux, 1992; Haettig et al., 2011). The deficits observed in contextual fear conditioning, but not OLM, might therefore suggest impairments in amygdala functioning. This possibility could be evaluated by performing cued-fear conditioning, a memory task requiring the amygdala that is independent of the hippocampus (Phillips and LeDoux, 1992). Although previous work using a similar CaMKIIα–tTA driver line demonstrates robust transgene expression levels in both the hippocampus and the amygdala, an important future direction would be to confirm amygdala expression of H3.3-HA in the tetO-H3.3-HA animals (Mayford et al., 1996). In addition to deficits in contextual fear memory, these animals also displayed deficits in motor learning. The rotarod task is linked to cortical and striatal function, and future studies should thoroughly evaluate H3.3-HA expression in these regions as well (Costa et al., 2004; Dang et al., 2006). A possible strategy to mitigate behavioral deficits would be to restrict transgene expression to a shorter window by altering the timing of doxycycline treatment, as is done with the fos-tTA driver line (Reijmers et al., 2007). Alternatively, we could instead utilize the Cre-dependent, double-floxed inverted orientation system combined with CaMKIIα-Cre mice, to virally express H3.3-HA selectively in excitatory neurons (Schnütgen et al., 2003). This would allow for more precise spatial specificity, as virus injections can be restricted to the hippocampus, and would allow for a shorter duration of transgene expression (Havekes et al., 2014).

The tagged H3.3 transgenic line is the second example of a tagged histone overexpression system developed in mice (Ito et al., 2014). Previous work has employed the tetracycline transactivator system to express a GFP-tagged histone H2B specifically in excitatory neurons of the forebrain (Ito et al., 2014). The overexpression of H2B-GFP was shown to produce marked consequences on chromatin architecture, perhaps through the steric interference of compacted heterochromatin structures (Ito et al., 2014). These structural changes were associated with alterations in gene expression at specific genomic loci as well as behavioral effects including hyperlocomotion, reduced nociception, and deficits in spatial memory and contextual- and cued-conditioning (Ito et al., 2014). Although it is unlikely that the nine amino acid HA tag would cause steric hindrance in a way that would dramatically alter chromatin architecture, it is possible that overexpression of H3.3-HA may cause chaperone dysregulation or alterations in baseline and activity-induced gene expression, both of which could contribute to the behavioral abnormalities observed here. These possibilities can be tested in future experiments using immunohistochemistry and qPCR-based methodologies.

There is growing interest in understanding the role of histone variant exchange in the brain and recently, the dynamic exchange of two histone variants in particular has been shown to contribute to long-term memory (Zovkic et al., 2014; Maze et al., 2015). Notably, histone variant H3.3 is dynamically deposited into the nucleosome in an activity-dependent fashion, helping to drive changes in gene expression required for synaptic connectivity and long-term memory (Michod et al., 2012; Maze et al., 2015). Because H3.3 is deposited in an activity-dependent fashion, this begs the question of whether a learning task may alter the localization of the tagged H3.3 in the genome. If this is the case, comparing changes in histone PTMs following learning may be confounded by differing genomic associations. This could be addressed by comparing ChIP-seq in transgenic animals after learning with control animals to define H3.3-HA localization across the genome. Additionally, ChIP-qPCR could be used in these mice to demonstrate “barcoding” of active regions of the genome following a learning event.

In summary, the tagged H3.3 transgenic mouse line provides a simple, adaptable tool to address the issue of cellular heterogeneity in neuroepigenetics. While excitatory neurons are a logical starting point for evaluating epigenetic changes during long-term memory consolidation, an advantage of using the tetracycline transactivator system is that it allows for substantial flexibility in terms of cellular specificity, as many cell-type specific tTA driver lines are available. Indeed, the tetO-H3.3-HA line could be combined with GFAP-tTA or fos-tTA lines to drive expression in astrocytes or recently-activated cells, respectively (Reijmers et al., 2007; Florian et al., 2011). In addition to its usefulness across cell types, we anticipate that this line could be employed to study the epigenome during spatial memory consolidation using the OLM task. Defining the changes in histone PTMs following learning is critical to understanding transcriptional regulation during long-term memory consolidation and may help to uncover novel epigenetic targets for future therapeutic benefit.

## Author Contributions

Transgenic mouse design by SGP and TA. Molecular characterization by AGM, SGP, and BAM. Behavioral studies conducted by AGM. Scoring of behavioral video by KMW. Data analysis and interpretation by AGM. Manuscript preparation by AM with editing by SGP, BAM, KMW, and TA.

## Funding

This research was supported by NIH R21 MH102679 to TA. AGM and SGP acknowledge funding from the Pharmacology Graduate Group Training Grant T32 GM008076.

## Conflict of Interest Statement

The authors declare that the research was conducted in the absence of any commercial or financial relationships that could be construed as a potential conflict of interest.
